The article "Drug-Induced Hepatotoxicity: Metabolic, Genetic and Immunological Basis" was published in 2014. Journal: Int J Mol Sci.

# Drug-Induced Hepatotoxicity: Metabolic, Genetic and Immunological Basis

**DOI:** 10.3390/ijms15046990

**Published:** 2014-04-22

**Authors:** Dolores B. Njoku

**Affiliations:** Departments of Anesthesiology and Critical Care Medicine, Pediatrics and Pathology, Johns Hopkins University, 1800 Orleans Street, Suite 6349, Baltimore, MD 21287, USA; E-Mail: dnjoku@jhmi.edu; Tel.: +1-410-955-2393; Fax: +1-410-502-5312

**Keywords:** drug induced liver injury (DILI), hepatotoxicity, pathogenesis

## Abstract

Drug-induced hepatotoxicity is a significant cause of acute liver failure and is usually the primary reason that therapeutic drugs are removed from the commercial market. Multiple mechanisms can culminate in drug hepatotoxicity. Metabolism, genetics and immunology separately and in concert play distinct and overlapping roles in this process. This review will cover papers we feel have addressed these mechanisms of drug-induced hepatotoxicity in adults following the consumption of commonly used medications. The aim is to generate discussion around “trigger point” papers where the investigators generated new science or provided additional contribution to existing science. Hopefully these discussions will assist in uncovering key areas that need further attention.

## 1. Introduction

Although nearly all classes of drugs can induce hepatotoxicity, drug induced liver injury (DILI) is a rare event. For the purpose of this review the term “drug” refers to commonly used medications. Since 1998 notable investigators clearly identified drug-induced hepatotoxicity as an endemic problem. To this end, Schiodt in 1999 [1], Temple and Himmel [2] as well as Ostapowicz in 2002 [3] in addition to Lee and Senior in 2005 [4], identified specific drugs and outcomes directly associated with drug-induced hepatotoxicity. As expected, these landmark discoveries in the population statistics of drug-induced hepatotoxicity as well as key discoveries in the area of pathogenesis of drug-induced toxicity produced even more questions about its metabolic, genetic and immunologic basis [5,6].

Despite lingering questions regarding key steps in the pathophysiology, most researchers agree that the etiology of drug-induced hepatotoxicity can be generally divided into two broad categories. The first category consists of direct hepatic injury or toxicity caused by the drug itself or by one of the drug metabolites. The second broad category is much more diverse. This category is mostly described as idiosyncratic. However in recent years, this category has been further divided into host-dependent or host-independent categories, where sometimes the divisions are not so clear. In the host-dependent category we find the genetic causes of drug-induced hepatotoxicity where metabolic causes are described either independently or associated with a genetic predisposition. In the host-independent category, immunologic causes are described; however, more and more these immune responses may have a genetic or even metabolic basis.

This review will cover papers that have addressed the metabolic, genetic and immunologic basis of drug-induced hepatotoxicity in adults. Children represent a unique group with respect to drug-induced hepatotoxicity and will be covered separately. Monoclonal antibodies as well as drugs utilized to treat HIV, infectious hepatitis or cancer have all been associated with hepatotoxicity. However, the complicated nature of their role in hepatotoxicity requires detail that is beyond the scope of this review. Hence, few drugs associated with HIV, hepatitis or cancer will be discussed in this review. The aim of this review is to generate discussion among toxicologists and immunologists and uncover key areas in the pathogenesis of drug-induced hepatotoxicity that need attention.

## 2. Metabolic Basis of Drug-Induced Hepatotoxicity

In the most basic sense, the purpose of drug metabolism is to facilitate excretion of a less polar drug through the formation of more polar metabolites. The resulting water soluble compound can be excreted from the body by the kidneys. In most cases Phase I metabolism through oxidation, reduction or hydrolysis by CYP450 enzymes produces the polar metabolites that are then made water soluble and available for excretion by Phase II metabolism via glucuronidation or sulphation. However, we cannot ignore the fact that activities of hepatic drug-metabolizing enzymes may be affected by expression of genes associated with these enzymes in addition to alterations in blood flow to the liver in normal and pathogenic states. In this section the role of metabolism in the pathogenesis of drug hepatotoxicity will be discussed.

In some cases, a drug or its metabolite may induce hepatotoxicity directly by gaining access to proximally located vulnerable hepatocytes. Acetaminophen is the most-well studied drug that is believed to use this mechanism. Direct hepatotoxicity of acetaminophen is dose-related that follows either one large single dose or a large cumulative dose of acetaminophen. The final pathway of hepatocyte injury is via binding of a toxic *CYP2E1*-derived metabolite, *N*-acetyl-*p*-benzoquinone imine (NAPQI), to subcellular organelles that induces necrosis or apoptosis [7]. Several other drugs are also capable of inducing dose-related hepatotoxicity that takes many forms. Direct hepatotoxicity from hepatocyte necrosis can occur following bromfenac, cyclophosphamide (direct injury to hepatic sinusoidal cells) or methotrexate [7]. Ischemic necrosis can be induced by cocaine, phencyclidine or niacin [7]. Steatohepatitis can be induced by amiodarone [7].

Metabolism takes center stage in the development of drug hepatotoxicity through the formation of directly toxic or reactive metabolites that exert their effect three possible ways. The first way involves direct injury to the hepatocyte by interfering with critical cellular functions. Metabolic activation of acetaminophen by CYP2E1 as an example leads to the formation of the toxic metabolite NAPQI. This much studied metabolite has a binding preference for intracellular organelles including the mitochondria [8]. In this site, through mechanisms that have not been completely elucidated, NAPQI triggers oxidant stress [9] which is believed to have a critical role in the development of hepatocyte necrosis [10] following the development of irreversible opening of mitochondrial membrane permeability transition pores [11]. Diclofenac is another NSAID capable of inducing direct hepatic injury at supratherapeutic doses through damage to subcellular organelles or through the formation of a benzoquinone imine metabolite in susceptible persons at normal doses [12]. Thus acetaminophen and NSAIDs may share common mechanisms of hepatotoxicity through metabolic activation and subsequent disruption of subcellular organelles.

The second way in which directly toxic or reactive metabolites may induce hepatotoxicity is through sensitization of the hepatocytes to cytokine-induced damage. An adaptation of this thought process has been utilized in the development of drug hepatotoxicity models where bacterial endotoxin, represented by LPS via TNF-α, in some cases, sensitizes the liver to injury [13]. Several models of hepatotoxicity ranging from moderate to severe necrosis have been demonstrated using this method. Hence, hepatotoxicity has been demonstrated following a single dose of LPS and a single dose of chlorpromazine [14], diclofenac [15], amiodarone [16], ranitidine [17], trovafloxacin or halothane [18]. Interestingly, the idea of two or more stimuli being required to induce an organ-specific immune response is a well-known mechanism that has been utilized in the development of animal models of autoimmunity. Hence these adapted models represent a step forward in toxicity modeling research since roles for cytokines in prior modeling were restricted to descriptive consequences of hepatotoxicity and not initiators of injury.

Reactive metabolites have an additional role in the development of hepatotoxicity through irreversible covalent modification of native proteins by reactive metabolites formed during drug metabolism, commonly known as haptenization. These covalently altered proteins subsequently promote immune recognition of these altered native proteins. In a susceptible host, this latter process triggers a cascade of cytokine driven immune reactions that culminate in hepatotoxicity. Since the bulk of the responses triggered by covalent modification are immune-mediated, they will be covered later in this review; however, in a classic review of drug reactions, immunologic and metabolic mechanisms were discussed together [19].

Notwithstanding, this review focuses on the contribution of intrahepatic metabolism to the development of hepatotoxicity, while, the contribution of extra-hepatic drug metabolism to the development of bioactive drug metabolites cannot be ignored. Sites of extra-hepatic metabolism include the small intestine, renal microsomes, lung parenchyma and plasma esterases. More investigations centered on the roles for these extrahepatic sites of metabolism in the development of hepatotoxicity are necessary in order to fully address the roles of metabolism in drug-induced hepatotoxicity.

## 3. Genetic Basis of Drug-Induced Hepatotoxicity

Prior to genome-wide association studies, genetics was believed to have a role in drug-induced toxicity. Bench researchers and physicians caring for patients looked for HLA haplotypes or other genetic markers that could help identify persons at risk for toxicity following certain drugs. Notable associations such as female sex and increased weight had been observed while individual variability in drug effect suggested differences in Phase I and Phase II enzyme expression that could explain some aspects of hepatotoxicity. Epigenetic responses had also been also implicated in hepatotoxic responses to drugs. This section will review current evidence for the genetic basis of drug hepatotoxicity, recognizing that in addition to the obvious role in identifying HLA haplotypes, genetics could have a role in the expression of Phase I and Phase II enzymes, cytokine expression or any enzyme system that has a role in the development of hepatotoxicity in response to drugs.

It is not surprising that HLA haplotypes have been targeted to study genetic associations of drug hepatotoxicity. In fact some of the strongest genetic associations have been made with HLA haplotypes and antibiotics associated with hepatotoxicity. In this way, amoxicillin-clavulinate was one of the earliest drugs identified where an HLA haplotype was associated with increased susceptibility to hepatotoxicity. Persons with HLA-DRB1 *1501-DRB5, *0101-DQB1 *0602 haplotype had approximately 10 times higher risk of developing hepatotoxicity following amoxicillin clavulinate when using genome wide association studies [20]. Earlier studies using the same technique determined that hepatotoxicity from flucloxacillin was 80 times more likely if a person expressed the HLA haplotye HLA B*5701 [21]. Interestingly other HLA types were associated with flucloxacillin but none was as strong as the HLA B haplotype association. More recent studies have performed genome wide association studies with the aim of identifying a genetic fingerprint that would help identify persons at risk; however, these investigators report the lack of statistically significant associations, highlighting the need for more widespread studies in order to aid the interpretation of their results.

The contribution of genetic expression of Phase I or II metabolic enzymes in the development of drug-induced hepatotoxicity presents an obvious mechanistic overlap in the basis of drug hepatotoxicity as organized it for this review. Although separated for the purposes of this review it is difficult to separate roles for by-products of metabolism from roles due to genetics when in some cases the amounts and forms of by-products can be genetically determined (Tables 1 and 2) [22]. In this way CYP2E1*1A has been associated with the generation of a toxic metabolite of anti-tuberculous drugs [23] in addition to the development of reactive oxygen species [24]. CYP2C8 has been associated with hepatotoxicity following the generation of toxic metabolites of diclofenac [25]. Additionally, differences in expression of CYP450 enzymes whether genetically determined or affected by disease processes should also be considered.

Phase II enzymes have long been associated with differences in metabolism; however, how differences in enzyme expression affect the development drug-induced hepatotoxicity has only been clarified in the last 10 years. To this end isoniazid has a well-known association with drug hepatotoxicity that is thought to be caused by multiple reactive metabolites. Two of these reactive metabolites acetylhydrazine and hyadrazine are known to be hepatotoxic and are metabolized by *N*-acetyl transferase. Persons with *N*-acetyl transferase 2 polymorphisims (slow metabolizers) have delayed detoxification of these toxic metabolites of isoniazid [26]. However, in addition to detoxification by *N*-acetyl transferase, glutathione *S*-transferase (GST) also has a key role in detoxification of reactive metabolites from isoniazid in addition to neutralization of reactive oxygen species. Hence, roles for glutathione *S*-transferase (GST) ranges from increased risk for mild hepatotoxicity from carbamazepine in persons who are GST theta 1 (GSTT1) null [27] to increased risk for significant hepatotoxicity from toxic isoniazid metabolites in persons who are GSTMI [28] or GSTT1 null [29] while GSTT1 GSTM1 double null persons are at increased risk for elevated ALT levels following troglitazone-induced mitochondrial injury via reactive oxygen species [30]. Lastly, isoniazid is not the only drug associated with hepatotoxicity where abnormalities in Phase II enzymes have been detected. Diclofenac hepatotoxicity has been associated with abnormalities in uridine-5′-diphosphate glucuronosyl tranferase 2B 7*2 where the mechanism of toxicity is believed to arise from increased formation of toxic metabolites [25].

Differences in expression of proteins associated with other aspects of drug disposition have been detected in patients with drug-induced hepatotoxicity. To this end, genetic differences in drug transporters have been detected in patients with drug-induced hepatotoxicity. In these situations, proteins such as multi drug resistance protein and bile salt export pump that are responsible for the excretion toxic products of drug metabolism in the bile have been associated with drug-induced hepatotoxicity. Diclofenac hepatotoxicity has also been associated with genetic abnormalities of multi-drug resistance protein [21].

The contribution of genetics in regulating immune reactions that promote drug hepatotoxicity is another mechanistic overlap with regards to the basis of drug hepatotoxicity. While we separated these mechanisms for the purposes of this review, it is difficult to separate roles for aberrant genetic expression of cytokines that affect immune responses from the roles of the cytokine in generating the immune response. In this regards, cytokines as immune regulators of drug hepatotoxicity have been studied with respect to interleukin (IL)-4, IL-6 and IL-10 and the drug diclofenac. In these mechanisms IL-4 is believed to promote immune responses to diclofenac metabolites that culminate in diclofenac hepatotoxicity [31] while IL-6 [31] and IL-10 [32] diminish anti-inflammatory responses that may prevent diclofenac hepatotoxicity.

Thus genetics offers unique insight with respect to the contribution of MHC haplotype in the pathogenesis of hepatotoxicity from certain antibiotics. However, with respect to enzymes or proteins that participate in metabolism, disposition and excretion of drugs associated with hepatotoxicity, it is difficult to separate roles of genetics from roles for direct toxicity of drugs or their metabolites to vulnerable hepatocytes. Additionally, it is nearly impossible to separate genetic effects from immunological effects of cytokines in some patients. It is our opinion that animal models of drug hepatotoxicity may allow us to tease out contributions of genetics from those of metabolism or immunology.

## 4. Immune Basis of Drug Hepatotoxicity

The immune basis for drug hepatotoxicity has been an area of development for the last 30 years. Encouraged by the popular “danger hypothesis”, landmark papers studying acetaminophen and halothane strongly suggested that covalent modification of self by reactive drug haptens triggered the loss of self-recognition [19]. Subsequently, immune cells whose primary role is to attack invading organisms or non-self, such as bacteria and possibly viruses, would then attack self. The ensuing immune responses would induce an immune-mediated hepatitis, antibodies to drug haptens as well as autoantibodies to self-proteins. Interestingly, prior to this immune shift in the thought process surrounding drug hepatotoxicity, most investigations centered upon mechanisms of hepatotoxicity triggered by inadvertent administration of excessive amounts of the inciting drug.

Drugs associated with an immune basis of drug toxicity are usually kept in the immuno-allergic or autoimmune category. Immune cells, cytokines and chemokines have all been investigated as mediators of drug hepatotoxicity. This section will review studies that address these components with respect to initiation or activation of the immune response with respect to what is known about drug hepatotoxicity. With regards to initiation, it is generally agreed that this occurs through antigen recognition by helper T cells in concert with key cytokines. Subsequently, effector mechanisms involving key cytokines and immune cells will be discussed.

No one is absolutely sure of the timing of immune cell activation in patients that would result in drug hepatotoxicity. Patients who have been sensitized to hepatotoxic drugs generally remain asymptomatic until the “perfect immune storm” occurs. Investigators generally agree that for the undesirable immune storm to occur, the patient must be sensitized while simultaneous activation of the innate immune system is occurring. This idea of “two hits” required for sensitization is a well-accepted mechanism originally described as critical to the development of organ-specific autoimmunity. Nonetheless, in toxicology, investigators have hotly discussed how these mechanisms can occur in toxicology mouse animal models while immunology models are not even discussed. This reviewer feels that all of these models contribute to the understanding of this process since for immune-mediated allergy, auto-allergy or even auto-allergic-toxicology to occur, there must be either a sensitization period. Moreover, the immune system must develop responses to drugs whose immunogenicity relies on their metabolites that induce novel antigens or relies on recognition of shared sequences that trigger native immune responses. Thus, complete understanding of this immune-mediated “idiosyncratic” hepatitis will require a diverse and multidisciplinary effort of toxicologists and immunologists.

The least well-studied immune-mechanism is the role of immune activation via T or B cells in the development of drug hepatotoxicity. To attempt to strictly address initiation of immune responses to covalently altered liver proteins, my lab first demonstrated immune-mediated hepatitis by covalently altering syngeneic cytosolic liver proteins with the trifluoroacetyl chloride (TFA) metabolite of halogenated volatile anesthetics and immunizing female BALB/c mice with this altered proteins emulsified in complete Freund’s adjuvant [33]. This model demonstrated hepatitis at 3 weeks consisting of neutrophils, macrophages, eosinophils and mast cells; however only mild elevations of liver transaminases were seen. In later studies hepatitis in these mice was followed for 12 weeks. Prior investigations in my lab also demonstrated a key requirement for IL-4 [34] as well as roles for CD4^+^ T cells in the initiation of this process using adoptive transfer. Additionally antibodies to TFA and CYP2E1 were demonstrated. The detection of antibodies in a model of immune-mediated hepatitis from drug haptens was an important step since patients who develop drug-induced hepatotoxicity, have antibodies to TFA and CYP2E1 in their sera; hence, this report concluded that these steps may represent the initiation of immune-mediated hepatitis and antibodies in response to drug haptens. Since the development of our model we have confirmed roles for immune activation triggered by IL-4 in patients by demonstrating CYP2E1 IgG4 autoantibodies in patients with anesthetic DILI [35–37]. Another study that clearly investigated the immunological role of IL-4 in the initiation of immune mediated hepatitis showed that IL-4 initiated and augmented hepatotoxicity following dicloxacillin [38] utilizing blocking antibody and recombinant IL-4, respectively. Together these studies demonstrated that T cell activation in an IL-4 environment initiates drug-induced hepatic inflammation and hepatotoxicity in animal models and most likely immune-mediated hepatotoxicity in patients. Most recently, my lab has shown critical roles for IL-6 and estrogen in the initiation and sex bias seen in our model [39]. Future investigations surrounding roles for additional cytokines, such as IL-6, are necessary in order to completely understand their role in the initiation of immune-mediated hepatic inflammation or injury as well as their role in the development of sex bias in drug-induced hepatotoxicity.

Other aspects of initiation of the immune response such as antigen presentation by dendritic cells are far less studied. Interestingly, a recent study elegantly showed that dendritic cell depletion worsened acetaminophen hepatotoxicity [40]. While in direct contrast to what is expected, this finding highlights complex roles for dendritic cells that may be affected by large doses of acetaminophen required to induce these hepatotoxicity models. Moreover, as in other models of acetaminophen hepatotoxicity where a rapid onset of injury is demonstrated following high doses of acetaminophen, expected roles for dendritic cells in antigen presentation and adaptive immune responses seem less likely.

Effector immune mechanisms involving cytokines have been more extensively studied in acetaminophen hepatotoxicity. In these studies the innate immune system expressing T-helper 1 (Th1) associated cytokines such as IL-6 may reduce hepatotoxicity [41,42]. Results from a recent study appear to directly contrast these prior studies. In the recent study Th1 associated cytokines namely TNF-α and IL-6 were described as pro-inflammatory (destructive) and augmented hepatotoxicity in C57Bl/6J mice when compared to BALBL/c mice while Th2 associated cytokines were described as anti-inflammatory (protective) [43]. These contrasting results from well-designed studies may have arisen from differences in animal housing, study design or endpoints measured. These off target effects as coined by Jaeschke may have significant roles in the development of contrasting outcomes when investigating effector Th2 mechanisms in acetaminophen hepatotoxicity [44]. More evidence for off target effects on study outcomes occurred in two well-designed studies investigating roles for IL-4 in acetaminophen hepatotoxicity. One study demonstrated a pathogenic role for IL-4 in the development of acetaminophen hepatotoxicity [45] while an earlier study clearly shows a protective role for IL-4 in this process [46]. Interestingly, these types of contrasting results are not limited to IL-4 or acetaminophen. Current studies show that cytokine effects in the pathogenesis of hepatotoxicity induced by one drug may not translate to other drugs known to induce immune mediated hepatotoxicity. Along these lines, prior studies in my lab associated IL-13, the effector cytokine for IL-4, with increased inflammation in our model of immune-mediated hepatitis triggered by halogenated anesthetic drug haptens [34] while other investigators clearly showed that IL-13 is hepato-protective in acetaminophen hepatotoxicity [47]. Additional investigations in patients with immune-mediated hepatotoxicity from various drugs may help to define the immunological role for these cytokines in effector mechanisms responsible for drug hepatotoxicity.

Recently T helper (Th)17 signaling via IL-17 has also been investigated in order to uncover effector immunological mechanisms of drug hepatotoxicity. IL-17 has been detected in the sera from patients with idiosyncratic liver injury [48]. However, animal studies demonstrate elevations in IL-17 in early time points following large doses of acetaminophen [49] or diclofenac [50]. This surprising finding could suggest sustained induction of IL-17 in this disease process: early in the initiation of the immune response in addition to during the effector period. Moreover, this early expression of IL-17 could suggest that innate immune cells such as invariant NKT cells or presently unidentified macrophages may be the source of IL-17 [51]. These vexing findings surrounding IL-17 may also serve a greater role. Detecting a cytokine burst in a time period generally thought to house innate responses may support the danger hypothesis where innate immune activation must occur. What is not clear, however, is whether or not this IL-17 response is an expected outcome following a very large dose of acetaminophen.

The bulk of studies investigations effector immune basis of drug hepatotoxicity have focused on immune cells such as neutrophils, Kupffer cells, macrophages or eosinophils by depleting these cells and determining the effect following high doses of drug. Neutrophils are the most common cell type discussed in the pathogenesis of drug hepatotoxicity. The most commonly discussed drug is acetaminophen. Neutrophils are early responders that migrate to areas of hepatocyte distress in response to immune signaling via inflammatory mediators, hepatocyte apoptosis or hepatocyte necrosis; however, their exact role in acetaminophen hepatotoxicity has been controversial [52]. Most investigators agree that neutrophils remove damaged hepatocytes or hepatocelluar debris [53] in animal models of hepatotoxicity; however, the relevance of this mechanism to the pathogenesis of acetaminophen toxicity in patients is not completely clear.

Neutrophils have also been discussed in the development of drug-induced hepatotoxicity with halothane. Neutrophils are believed to directly mediate liver injury following intraperitoneal halothane [54]. A similar role for neutrophils was suggested following halothane in another mouse model [18]. A recent study has challenged the role of neutropils in hepatotoxicity following intraperitoneal halothane. This study demonstrated that hepatotoxicity was unaffected following immunologic depletion of neutrophils by anti-Gr-1 [55]. Interestingly, my lab previously demonstrated significant neutrophilic hepatitis induced by allergic responses to native liver proteins covalently altered by the trifluoroacetyl chloride metabolite of halothane and other halogenated volatile anesthetics [33]; however, only mild to moderate elevations in AST were seen after 12 weeks following induction of hepatitis. Hence these studies suggest that similar to acetaminophen, neutrophils may be present following a large dose of intraperitoneal halothane; however, whether or not these neutrophils contribute to the development of hepatotoxicity is controversial. Alternatively, neutrophilic inflammation may occur in response to damaged hepatocytes either from hepatotoxic drug administration or autoimmune attack triggered by sensitization to self-proteins.

Roles for Kupffer cells and infiltrating macrophages have been addressed in models of halothane and acetaminophen hepatotoxicity. Early detection of trifluoroacetylated adducts in Kupffer cells from guinea pigs exposed to halothane by inhalation identified these cells as possible key players in the development of halothane hepatotoxicity through antigen presentation of covalently altered proteins [56]. Subsequent investigators suggested a toxic role for Kupffer cells in the pathogenesis of hepatotoxicity following intraperitoneal halothane in addition to poly IC by demonstrating lowered ALT levels following Kupffer cell or NK cell depletion [57]. In this subsequent study ALT levels in the Kupffer cell depleted mice were similar to mice that developed hepatotoxicity following intraperitoneal halothane without poly IC. Hence, the authors suggested that Kupffer cell depletion in the face of viral illness mimicked by Poly-IC could be a scenario that affects patients. Prior studies in my lab show decreased Kupffer cells associated with increased immune-mediated hepatitis; however, we concluded that Kupffer cells have a protective role in immune-mediated hepatitis [33]. These divergent roles for Kupffer cells in halothane hepatotoxicity may reflect differences in the formulation of these models where in the former hepatotoxicity is clearly demonstrated following intraperitoneal halothane [57], while the latter clearly demonstrates autoallergic responses following sensitization by drug haptens [33].

Many investigators agree that Kupffer cells have a directly protective role in the pathogenesis of hepatotoxicity following acetaminophen utilizing models of Kupffer cell depletion [58]. A combined protective role for Kupffer cells and infiltrating macrophages was recently described following acetaminophen hepatotoxicity; however, this role rested in hepatic regeneration where separate depletion of these cells reported no significant effect of these cells on hepatotoxicity [59]. In contrast to these findings, another study demonstrated that while Kupffer cells may protect the liver, they may impair the lung following toxic doses of acetaminophen [60]. Hence additional roles for Kupffer cells in other organs should be considered when investigating toxicity of a drug with the ability for systemic immune derangements.

Infiltrating macrophages have also been investigated in the pathogenesis of drug hepatotoxicity. Recent studies clearly show that macrophages can have essential roles in the resolution of injury. Alternatively activated macrophages stimulated by IL-10, IL-4 or TGF-beta reduce inflammation and stimulate hepatic regeneration and repair [61,62]. Additionally, prior studies demonstrated that stem cell-derived tyrosine kinase receptor (STK) signaling on macrophages may down regulate inflammation through alternative activation of macrophages [63].

While other cells can be controversial, most investigators agree that eosinophils should have a role in immune-mediated hepatotoxicity. However, few studies identify eosinophils in models of drug-induced hepatotoxicity while eosinophils have been identified following the induction of T cell inflammation and hepatotoxicity with concanavalin A. My lab clearly identified eosinophils in a model of drug-hapten hepatitis which suggested to us that we had developed a model of immuno-allergic hepatic inflammation [33]. However, a recent study clearly demonstrated that eosinophils have a critical role in promoting the hepatic destruction following intraperitoneal halothane [55]. Thus, while classical roles for eosinophils are expected in the development of allergy to drug haptens, they may have a direct role in the development of hepatotoxicity following intraperitoneal halothane.

Roles for chemokines were recently reviewed in the development of hepatotoxicity [64]. Chemokines work locally in concert with cytokines and cells as immune-modulators of drug hepatotoxicity. The promotion of hepatotoxicity or hepato-protection depends on the chemokine, its receptor, the drug studied and sometimes even the cell affected. In this way macrophage recruitment in acetaminophen toxicity is promoted through CCL2 and its receptor CCR2 while CXCL8 and CXCL9 induce protective T cell responses in acetaminophen hepatotoxicity [64] as well as hepatic inflammation from drug haptens [65]. Because of the enhanced local responses in the liver, chemokines may offer promise for specific therapies in drug hepatotoxicity.

## 5. Conclusions

In conclusion, this review focused on studies surrounding drug hepatotoxicity where genetic, metabolic and immune mechanisms were investigated. While some studies addressed these areas separately with respect to drug hepatotoxicity, clear mechanistic overlap exists. Thus understanding mechanisms of drug hepatotoxicity will require a concerted and diverse effort between immunologists and toxicologists.

## Figures and Tables

**Table 1.** Genome-Wide Association Studies (GWAS) Showing Significant Roles for *Cytochrome P450* Genes. Reproduced with permission from Daly, A.K. [22].

Subject of study	Significant CYP gene
Warfarin dose requirement	*CYP2C9* and *CYP4F2a*
Acenocoumarol dose requirement	*CYP2C9* and *CYP4F2a*
Response to clopidogrel	*CYP2C19*
Smoking behavior	*CYP2A6b*
Caffeine intake	*CYP1A2c*

**Table 2.** Polymorphisms in Cytochromes P450 Relevant to Drug Metabolism and Their Functional Importance. Reproduced with permission from Daly, A.K. [22].

Gene	Common variant alleles	Functional effect
*CYP1A2*	CYP1A2*1F	High induced activity

*CYP2A6*	CYP2A6*2 and *4	Absence of activity
	CYP2A6*1X2A and *1X2B	High activity

*CYP2B6*	CYP2B6*2, *5 and *6	?Decreased activity

*CYP2C8*	CYP2C8*2, *3 and *4	?Decreased activity
	CYP2C8*5	Absence of activity

*CYP2C9*	CYP2C9*2 and *3	Low activity
	CYP2C9*6	No activity

*CYP2C19*	CYP2C19*2 and *3	No activity
	CYP2C19*17	High activity

*CYP2D6*	CYP2D6*3, *4, *5 and *6	No activity
	CYP2D6*10 and *17	Low activity
	CYP2D6*1XN and *2XN	High activity

*CYP3A5*	CYP3A5*3	No expression
